# Online Loan Default Prediction Model Based on Deep Learning Neural Network

**DOI:** 10.1155/2022/4276253

**Published:** 2022-08-08

**Authors:** Baodong Li

**Affiliations:** School of Statistics and Big Data, Henan University of Economics and Law, Zhengzhou 450046, Henan, China

## Abstract

With the rapid development of Internet loans and the demand for Internet loans, Internet-based loan default prediction is particularly important. P2P online lending is based on Internet technology. With the popularization of personal PCs and mobile terminals, the borrower's financing cost has been reduced to a large extent, and the efficiency of the borrower's capital utilization has also been improved to a considerable level. Making full use of the existing data of the online lending platform, integrating third-party data, and predicting the default behavior of users are the major directions of future development. This paper mainly studies the network loan default prediction model based on DPNN. This paper first analyzes the problems and risks of the P2P online lending platform, then introduces the principle and characteristics of BPNN in detail, and determines the credit risk rating process for online lending based on BPNN. With the help of data analysis and processing software, after cleaning and variable selection of credit customer data provided by lending clubs, a set of corresponding online lending default risk assessment models are established through BPNN. This paper simulates the network loan default assessment model of the BPNN model and compares it with the support vector machine and regression model. The experimental results show that the highest accuracy rate of the BPNN model is 98.01% and the highest recall rate is 99.82%, which is better than the other two models; the AUC value of BPNN is 0.79, which is significantly higher than that of support vector machine and regression model. The above results show that the online loan default prediction model based on DPNN has high application value in practice. Predicting the probability of customer default risk in advance will help reduce the risk of P2P companies and lenders, improve the competitiveness of P2P lending institutions, and promote the development of domestic P2P platforms to be more stable.

## 1. Introduction

Traditional financial institutions have high thresholds, low returns, and long investment cycles, making investors continue to seek new flexible, high-yield, and low-amount investment channels. At the same time, due to the imperfect personal credit information system in my country and the slow construction of credit information, some “good” funders cannot obtain funds from traditional financial institutions, resulting in low threshold and convenient operation. Deep learning is to learn the inherent laws and representation levels of sample data, and the information obtained during these learning processes is of great help to the interpretation of data such as text, images, and sounds. *P2P platform*. Peer-to-peer lending (P2P) is an intermediary platform that provides online information matching and auditing services for borrowers and lenders. Based on the P2P platform, lenders and borrowers openly lend and transfer money online [1]. The needs of investors and capital demanders have provided fertile soil for P2P development, which has greatly promoted the rapid growth of the P2P online lending platform. At the same time, P2P lending has become an important part of my country's financial market, playing an irreplaceable role in meeting the market's investment and financing needs and promoting the diversified development of the financial market. However, the P2P platform lacks financial management and risk prevention and control capabilities and cannot accurately and effectively assess the credit status of borrowers, resulting in a large number of bad debts on the P2P platform [2].

The development environment of China's P2P industry is not optimistic. It is particularly important to establish a sufficiently sound default prediction system and to accurately remind participants of default predictions for the healthy development of the P2P industry. Many experts have made outstanding contributions in the field of personal credit evaluation and created many valuable methods. Among them, several classic traditional credit rating methods mainly include *z*-rating model, regression analysis, and discriminant analysis. On the basis of ratio analysis, Yusuf discusses the multiobjective optimization model and establishes a multiobjective credit evaluation model in combination with the objective programming method. Then, his model is only applicable to the commercial banking environment and does not consider the applicability of online lending platforms [3]. Grace built a logistic regression model and a radial basis function model to predict defaults in commercial bank personal loan data. By comparing the two modes, we can clearly see that each mode has its own advantages and disadvantages. The overall accuracy of the logistic regression model is higher than that of the radial basis function model, but the efficiency of the radial basis function model is more effective in determining the potential default risk of users [4]. Jan builds a decision forest model based on association adaptation and compares it with a climbing decision tree model and a random forest model. The results show that the CADF model is more suitable for credit risk prediction, and the prediction accuracy of the model is better than other models. However, the performance of this model cannot be compared with the NN model [5].

This paper uses BP neural network (BPNN) to establish a network loan default prediction model. Relying on certain principles, select indicators and create a prediction system for the default of borrowers in the current market P2P industry and design a neural network prediction model on the basis of the BP algorithm. Compared with traditional machine learning processing a large amount of data, the BPNN loan default prediction model established in this paper has a high accuracy rate, which can be better than the actual use of online loan platforms, further improving the prediction accuracy rate, providing high-quality borrowers, and attracting loans are of great significance.

## 2. Establishment of P2P Network Lending Platform and Default Prediction Model

### 2.1. Problems and Risks of P2P Online Lending Platform

The generation of P2P online lending mainly refers to the financial model in which individuals provide small loans to other individuals through third-party platforms on the premise of charging a certain fee.

#### 2.1.1. P2P Online Lending Risk Definition

*(1) P2P, i.e., Person-to-Person (Partner-to-Partner)*. Also known as peer-to-peer online lending, it is a private microlending model that aggregates small funds and lends them to people in need of funds.

With the emergence of P2P trading platforms, the risks of many P2P platforms have also increased. Among them, the risks from P2P platforms mainly include the following aspects: operational risk. On the one hand, some platforms are essentially so-called Ponzi schemes, that is, empty-handed wolves, borrowing new ones to repay the old ones and repaying the principal and interest of the front-end investors with the money of the investors behind them. There are no physical borrowers at all. On the other hand, due to poor management and low level of risk control, some platforms often have overdue and bad debts.

*(2) Risk of Capital Pools and Illegal Misappropriation of Funds*. A P2P platform should generally be a peer-to-peer connection between borrowers and borrowers [6]. At this time, the customer's account funds are easily misappropriated illegally. These misappropriated funds are used by the platform itself, or for other investments, or overdue project advances, or to make up for bad debts.

*(3) Product Alienation Risk*. The second tender is the loan subject with immediate repayment after the full tender, which has the characteristics of short term and high income. It is designed to familiarize new customers of the platform with the rules and attract investors. There is no real borrower behind it. But there are also platforms that use this as a tool to expand the scale of transactions, improve website rankings, and reduce bad debt rates, thereby winning the trust of investors. There are also some platforms that absorb funds in seconds after illegal possession, and a large amount of funds abscond.

*(4) Cyber Technology Risks*. The business of the P2P platform depends on the Internet. The Internet brings convenience and speed to the P2P industry, but it also brings many problems [7]. Due to the lack of strength of many platforms, limited capital and technical investment, and inadequate system construction, security protection, and information maintenance, the platforms are often hacked or information is leaked.

*(5) Spill Risk*. After an accident occurs on a P2P platform, risk spillover is prone to occur, which not only affects the financial system. In the past, the risk events of some P2P platforms involved many private enterprises. The broken capital chain makes it difficult for these enterprises to repay bank loans, resulting in an increase in bank nonperforming assets [8].

The risk from the borrower is mainly manifested as credit risk, that is, the borrower defaults or defaults, which often occurs in P2P network lending. The characteristics of the P2P industry determine that most of its customers are high-risk borrowers. At the same time, due to the poor review of online lending platforms and asymmetric information, platforms and lenders cannot accurately judge the true situation and repayment ability of borrowers, resulting in frequent defaults of borrowers [9, 10].

The advantages of P2P online loans are fast loan, the same day; simple approval procedures; higher annual interest rates on online loan platforms; and no mortgage and guarantee.

#### 2.1.2. P2P Online Lending Platform Risk

P2P is a kind of Internet financial product. It is a private microloan, an online credit platform, and related financial management behaviors and financial services with the help of the Internet and mobile Internet technology. The risks are as follows:

*(1) Information Asymmetry*. Since borrowers and lenders are usually strangers from different regions, lenders cannot fully understand the borrower's basic information, economic status, use of funds, and other information, nor can they confirm the authenticity of such information. In addition, due to the imperfect credit reporting system, some borrowers will forge personal information to conduct malicious breach of contract and fraud, thus causing huge losses to online lending platforms and borrowers.

The borrower's credit default risk is high. Traditional financial institutions are still the first choice for high-quality borrowers, which are not only safe and reliable but also have much lower interest rates than P2P loans. Therefore, most of the P2P customers are individuals and small and microenterprises who have difficulty in obtaining funds in the traditional financial system. Their credit level and repayment ability are relatively poor, and their default risk is high. The platform's higher interest rates, in turn, increase the repayment pressure on borrowers. In addition, my country's social credit system is not perfect, information is not effectively shared, and the risk of default is greatly increased [11].

Industry entry barriers are low. In the early days, the access conditions of China's online lending platforms were mainly limited by registered capital, and other requirements were very low or not. In the early years, a P2P platform could be established with only a few hundred thousand yuan. There are many illegal enterprises, and there are very few truly high-quality platforms. In addition, many P2P platform entrepreneurs do not have professional financial and risk control knowledge, and even some platforms do not have a fixed office space and risk control department, which limits the overall quality of China's online lending platforms.

The supervision is weak, and the system is not perfect. As an emerging industry, P2P network lending was not regulated by institutions in the early days. The lack of relevant regulations and systems makes the internal operation of the industry chaotic, various platforms flood into disasters, and problematic platforms are frequently exposed [12]. In recent years, the China Banking Regulatory Commission has successively issued relevant regulations and management measures to regulate and rectify the P2P industry, but the regulatory system is still not perfect, and relevant policies need to be further implemented and implemented. For the risks of P2P online lending, the flow chart of P2P online lending is shown in Figure 1.

### 2.2. Detailed BPNN

#### 2.2.1. Overview of Neural Networks

NN is an artificial neural network (ANN). It can also be called a Neural Network (NN) in the sense of not causing confusion. As the name suggests, the NN model imitates the nervous system of animals, transmits information between neurons, and responds to external stimuli. Both BP neural network and deep learning belong to one of the neural networks. Generally, neural network refers to artificial neural networks other than BP neural network and deep learning. BP neural network is the top representative of artificial neural networks.

A typical neural network consists of three parts: structure, activation function, and learning rules [13]. The structure is the composition of the NN, what variables are there, such as the connection weights and excitation values between neurons, and the relationship between these variables; the activation function is a function that determines how neurons respond according to the activity output of other neurons, generally related to connection weights between neurons; and learning rules determine how connection weights are adjusted and optimized during training [14].

#### 2.2.2. BPNN Principle

NN is a network structure formed by some simple components connected to each other through complex layers. It can simulate how the nervous system works to reflect specific things. In this complex network, it is generally necessary to artificially define multiple input and output items. There are usually one or more hidden items between the input and output items [15].

Depending on the number of hidden layers, there are single-hidden-layer NNs and double-hidden-layer NNs. Generally speaking, increasing the number of hidden layers can improve the learning ability of the entire neural network, but at the same time, it will greatly increase the learning time and reduce the efficiency. In general, the hidden layer will not exceed two layers [16, 17]. As shown in Figure 2, BP is the structure diagram of NN.

The BP neural network is the most basic neural network, its output is forward-propagated, and the deviation is back-propagated.

The mathematical model expression of BPNN is as follows:

(1) $$\begin{array}{c} y_{i}=f\sum_{j=1}^{n}\omega_{ij}x_{j}+\theta_{j}. \end{array}$$

BPNN is also called logsig, Tansig and purelin. The input values of these three transfer functions can be arbitrary, which ensures the comprehensive adaptability of the model in application. Different transfer functions have different output intervals. Different transfer functions can be chosen to handle different problems to guarantee the effectiveness of the overall NN model.

In fact, the learning process of BPNN is to simulate the learning process of biological neural network. In the initial stage of biological learning, more NN learning process is equivalent to conditioned reflex, which requires repeated training to form stable feedback results. The learning process of BP NN also requires repeated training. First, calculate the error of the output layer and then use this error to calculate the error of the previous layer (layer by layer). In this way, the error of each layer in the NN can be gradually obtained. For the update of the weights and thresholds of NN, we need to calculate the partial derivatives. By continuously adjusting the network weights and thresholds, the gradient search technology is used to calculate the weights and thresholds of the NN using the error backpropagation algorithm. The modified weights and thresholds are calculated iteratively in order to minimize the mean squared error between the actual and expected outputs computed by the network [18, 19].

During the training of the NN, there is no need to understand the mathematical relationship between the input and output results. NNs are trained from a large amount of input and output data with known correspondences. Some rules are formed naturally during training. When given an input value again, the result closest to the expected value can be obtained by network calculation [20].

#### 2.2.3. Characteristics of BPNN and P2P Online Lending

Characteristics of P2P online lending are as follows: direct and transparent, the lender and the borrower directly sign a personal-to-person loan contract; credit screening, the lender can evaluate and select the credit of the borrower; and risk dispersion, the lender distributes funds to multiple borrower object.

BPNN draws on the advantages of biological neural network, so it has the following characteristics:

*(1) High Degree of Parallelism*. BPNN is parallel in structure, so it can process a large amount of information in the network. For many problems with unclear causal relationships, the parallel processing capability of this massive amount of information can make the final analysis results more accurate.

*(2) Distributed Storage and Fault Tolerance*. BPNN is carried out through weights. For complex problems of analysis, through the training process of NN, rules and experience are accumulated and all are distributed and stored in the weights of the whole NN. Even if the stored information is lost, the system can still be analyzed to make it fault-tolerant.

*(3) Self-Learning, Self-Organization, and Self-Adaptation*. BPNN is reflected in the variability of its structure. The weights of each neuron are adjusted by training self-organization to adapt to changes in external conditions. By learning a large amount of data, NN can adapt to the solution of various problems under the model and has a certain ability to adapt to the data.

*(4) Global Nonlinear Output*. In general, the entire operation process of BPNN is the joint action of all neurons to generate nonlinear output so that the output of BPNN will not be disturbed by individual factors. The results of this network's analysis are global.

### 2.3. Establishment of BPNN P2P Online Loan Default Prediction Model

Aiming at the classification and prediction of credit default of loan customers on the P2P online loan platform, the backpropagation algorithm (BP algorithm) of the multilayer perceptron is used to establish a three-layer NN structure. Among them, the number of nodes in each layer is 243, processing and analyzing the characteristics of the loan customer data of the online loan platform, and training the NN model.

In the selection of the hidden layer, some scholars have proved that when the hidden layer has enough neurons, the NN structure of a single hidden layer is often better than the NN structure of the multilayer hidden layer neural structure and can approximate any continuous function infinitely. Therefore, in order to make the network structure simpler, this paper adopts a three-layer BPNN, that is, there is only one hidden layer. However, there is no unified and feasible theoretical support for the selection of hidden nodes, and it is usually determined with reference to the experience of experts and the process of multiple network training and optimization.

#### 2.3.1. Algorithm Details

Input: data set, learning rate, multilayer neural network architecture; output: a trained neural network; initialization weights and biases *T* are randomly initialized between −1 and 1 (or whatever), per unit has a bias; for each training instance *X*, perform the following steps:

(1) According to the NN model, the following formula formula (2) can be obtained:
  (2) $$\begin{array}{c} o_{j}=\sum_{i}w_{ij}x_{i}+\theta_{j}. \end{array}$$
From hidden layer to output layer, formula (3) is as follows:
  (3) $$\begin{array}{c} o_{k}=\sum_{j}w_{jk}o_{j}+\theta_{k}. \end{array}$$
Two formulas are summed up as follows:
  (4) $$\begin{array}{c} I_{j}=\sum_{i}w_{ij}o_{i}+\theta_{j}. \end{array}$$
Define the following formula:
  (5) $$\begin{array}{c} f\left(x\right)=\frac{1}{1+e^{-x}}. \end{array}$$
The output of each layer is as follows:
  (6) $$\begin{array}{c} o_{j}=\frac{1}{1+e^{-I_{j}}}. \end{array}$$
(2) According to the error reverse transmission, for the output layer, *T* k is the true value and O *k* is the predicted value; the formula is as follows:
  (7) $$\begin{array}{c} Err_{i}=o_{k}\left(1-o_{k}\right)\left(T_{k}-o_{k}\right). \end{array}$$

For the hidden layer, the formula is as follows:

(8) $$\begin{array}{c} {\text{Err}}_{i}=o_{j}\left(1-o_{j}\right)\sum_{k}{\text{Err}}_{k}w_{jk}. \end{array}$$

Updating the weights and *l* is the learning rate.

(9) $$\begin{array}{c} \Delta w_{ij}=\left(l\right){\text{Err}}_{i}o_{j},\\ w_{ij}=w_{ij}+\Delta w_{ij}. \end{array}$$

Bias update is given by the following formula:

(10) $$\begin{array}{c} \Delta \theta_{j}=\left(l\right){\text{Err}}_{i},\\ \theta_{j}=\theta_{j}+\Delta \theta_{j}. \end{array}$$

In NN, the activation function is used for linear combination calculation, which realizes the operation of the hidden layer. At the same time, since the classification method in this paper is binary classification, the sigmoid function is also used in the output layer to control the returned output value within the range of [0, 1].

## 3. Simulation Experiment of Online Loan Default Prediction Model Based on Deep Learning Neural Network

### 3.1. Simulation Experiment Data Source

The data in this article come from the famous P2P platform lending club. Lending club publishes personal loan default recovery information on its official website. This paper selects more than 30,000 loan account information and corresponding default recovery information within six months as the research data set.

### 3.2. Simulation Experiment Plan

This paper compares the prediction effect of BPNN, support vector machine, and regression model on loan application data of P2P platform; compares the prediction effect of BPNN under different number of hidden layer nodes; and finds out the best algorithm model based on loan data.

As shown in Table 1, it is the experimental platform of the program developed in this paper.

### 3.3. Evaluation Standard

The most widely used model evaluation methods are still precision and recall. The call rate is defined as the correctly predicted positive samples out of the total sample. As a classic evaluation standard, the formula is as follows:

(11) $$\begin{array}{c} P=\frac{\text{TP}}{\left(\text{TP}+\text{FP}\right)},\\ R=\frac{\text{TP}}{\left(\text{TP}+\text{FN}\right)}. \end{array}$$

## 4. Simulation Results of Online Loan Default Prediction Model Based on DPNN

### 4.1. Evaluation Effect of Different Hidden Nodes

The records of precision and recall are shown in Figure 3.

According to the data shown in Figure 3, as the number of hidden layer nodes increases, the accuracy of the algorithm also increases first. Then, when the hidden layer contains 9 nodes, the accuracy of BPNN reaches a higher level. This paper selects the BPNN evaluation model with 9 hidden nodes for analysis and experiment.

### 4.2. Evaluate the Effect of the Experiment

As shown in Table 2 and Figure 4, the accuracy of the BPNN model in credit evaluation is significantly better than that of the support vector machine and the regression model. Among the three sets of data, the highest accuracy rate of the support vector machine is 92.81%, and the highest recall rate is 98.54%; the highest accuracy rate of the regression model is 93.27%, and the highest recall rate is 98.61%; the highest accuracy rate of the BPNN model is 98.01%, and the highest recall rate is 99.82%. It can be seen that the BPNN model is better than the other two prediction models in terms of accuracy and recall.

### 4.3. Prediction Error for Different Model Samples

As shown in Table 3 and Figure 5, the mean squared errors of the three models on the six sets of predictions are shown. It can be seen that the MSE value of the BPNN model is always lower than that of the support vector machine and the regression model, indicating that the BPNN model improves the accuracy of the default prediction.

As shown in Table 4 and Figure 6, the differences between the true and predicted values of the default loss rates for BPNN, SVM, and regression models are shown. Most of the test set prediction difference is below 0, indicating that the model tends to overestimate the recovery rate, that is, underestimate the default loss rate. However, the difference between the prediction results of the BPNN model and the real value is smaller, and it is closer to the real recovery rate.

### 4.4. User Prediction Results

This paper sorts the default probabilities of all topics in descending order and divides them into ten groups, each labeled 1–10 as shown in Figure 7. The lower the number of groups per group, the higher the user's risk of default. At the same time, this paper introduces the commonly used improvement table in the scorecard to analyze the actual performance of each group of users and uses the ratio of the marginal default rate and the cumulative default rate relative to the entire group as the evaluation indicators.

### 4.5. Comparison of Prediction Results for All Models

As shown in Table 5 and Figure 8, after calculating the ROC curves of FPR and TPR, the AUC areas under the ROC curves of the three models were calculated to further compare the classification effects of the three models. It can be seen that the AUC value of BPNN is 0.79, which is significantly higher than that of the SVM and regression model. Based on the above results, we can conclude that the evaluation effect of the BPNN model is better than that of the traditional machine learning model.

## 5. Conclusion

With the development of Internet technology, Internet ideas and new concepts have also entered the financial industry, thus giving birth to the Internet financial industry. Among them, a new form of loan—P2P network lending—not only meets the needs of personal lending but also meets the financing needs of small and medium-sized enterprises, increasing the investment channels for investors. In order to ensure the sustainable development of the P2P online lending industry and provide safer and more timely services for more borrowers and investors, this paper analyzes and studies relevant domestic and foreign literature and mature P2P online lending platforms and understands the mainstream P2P online freight. Domestic and foreign business models, and with reference to commonly used credit risk assessment models, combined with the historical transaction data of Wallet Finance to establish risk assessment and prediction models.

This paper mainly studies the network loan default prediction model based on deep learning neural network (DPNN) and establishes the network loan default prediction model through BPNN. This paper compares the effectiveness of deep learning BPNN and traditional machine learning in evaluating default probabilities when dealing with large amounts of data. Due to its special network structure, it not only has the best evaluation effect but also can learn adaptively, which can effectively evaluate the risk of default probability and reduce the cost of risk management.

BPNN model is significantly higher than that of other traditional machine learning models, and it can automatically learn from data, reducing the time and cost of manually designing feature variables, and can better predict the default probability of loans. Therefore, the online loan default risk assessment model framework established in this paper has certain advantages in the field of loan risk assessment and management in the online loan industry and can help online loan companies to better manage their online loan default problems.

## Figures and Tables

**Figure 1:** Flow chart of P2P online loan.

**Figure 2:** BPNN structure diagram.

**Figure 3:** Accuracy of different hidden nodes.

**Figure 4:** Evaluation results of the three models.

**Figure 5:** Out-of-sample forecast mean squared error time series for three models.

**Figure 6:** Out-of-sample forecast error time series for three models.

**Figure 7:** The distribution of lift index for each group.

**Figure 8:** Comparison of prediction results of all models.

**Table 1:** Experimental platform name parameter table.

Environmental	Name	Parameter
Hardware environment	CPU	Intel(R) Core i7-10700k 3.8 GHz 8 cores
	Graphics processor	Nvidia GeForce RTX 3080
	Memory	16 GB
	Hard disk	Western Digital Black SN750 500G Solid State Drive

Software environment and tools	Operating system_	Ubuntu 16.04
	Programming languages and tools	Python 3.6.7
		Anaconda, scikit-learn, TensorFlow

**Table 2:** Evaluation results of the three models.

Data set	Support vector machines		Regression model		BPNN	
	Accuracy (%)	Remember (%)	Accuracy (%)	Remember (%)	Accuracy (%)	Remember (%)
One	91.23	97.64	92.14	98.05	95.42	99.18
Second	92.07	97.96	92.73	98.37	96.74	99.42
C	92.81	98.54	93.27	98.61	98.01	99.82

**Table 3:** Out-of-sample forecast mean squared error time series for three models.

	One	Second	C	D	Second	F
Support vector machines	0.0037	0.0035	0.0031	0.0027	0.0029	0.0034
Regression model	0.0032	0.0029	0.0026	0.0022	0.0024	0.0028
BPNN	0.0027	0.0025	0.0021	0.0012	0.0018	0.0023

**Table 4:** Out-of-sample forecast error time series for three models.

	One	Second	*C*	*D*	Second	*F*
Support vector machines	−0.013	−0.018	0	−0.028	−0.036	−0.038
Regression model	−0.006	−0.012	0.004	−0.019	−0.030	−0.028
BPNN	0.007	−0.009	0.015	−0.01	−0.024	−0.006

**Table 5:** Comparison of prediction results of all models.

	Support vector machines	Regression model	BPNN
Area under the curve	0.68	0.72	0.79
Prediction accuracy of normal loans	71.57%	75.41%	81.34%
Predictive accuracy of defaulted loans	75.42%	80.07%	84.05%

## Data Availability

No data were used to support this study.
